RETRACTED

# Prediction of the Collapse of Necrotic Femoral Head by CT and X-Ray Examinations before Hip Replacement Based on Intelligent Medical Big Data

**DOI:** 10.1155/2021/9971236

**Published:** 2021-12-22

**Authors:** Yongwei Shang, Jianjie Xu, Ting Zhang, Zhihui Dong, Jiebing Li, Weidong Bi, Zhe Xie

**Affiliations:** ^1^The Second Department of Orthopedics, The People Hospital of Shijiazhuang, Shijiazhuang 050000, China; ^2^Department of Orthopedic Surgery, Third Hospital of Hebei Medical University, Shijiazhuang 050000, China

## Abstract

It was to explore the effect of the CT and X-ray examinations before the hip replacement to predict the collapse of the necrotic femoral head under the classification of medical big data based on the decision tree algorithm of the difference grey wolf optimization (GWO) and provide a more effective examination basis for the treatment of patients with the osteonecrosis of the femoral head (ONFH). From January 2019 to January 2021, a total of 152,000 patients with ONFH and hip replacement in the tertiary hospitals were enrolled in this study. They were randomly divided into two groups, the study sample-X group (X-ray examination results) and based-CT group (CT examination results)—76,000 cases in each group. The actual measurement results of the femoral head form the gold standard to evaluate the effect of the two groups of detection methods. The measurement results of X-ray and CT before hip replacement are highly consistent with the detection results of the physical femoral head specimens, which can effectively predict the collapse of ONFH and carry out accurate staging. It is worthy of clinical promotion.

## 1. Introduction

The osteonecrosis of the femoral head (ONFH) is a common and multiple orthopedic disease in the clinic. The main clinical manifestations are hip pain and dysfunction [1–3]. By the occurrence mechanism, it is known that ONFH disease is a progressive pathological evolution process [4], and the clinical treatment experience shows that ONFH disease is difficult to treat. If patients with ONFH cannot get effective treatment for a long time, it will lead to the collapse of the femoral head and cause inflammatory lesions, which have a great impact on the hip joint [5]. In the treatment, whether the operation method is symptomatic will have a greater impact on the treatment effect [1]. At present, there is no general method that can directly cure the different stages, types, and necrotic volume of the femoral head. According to the stage of ONFH disease, mastering the indications of surgical treatment is the main method, especially for palliative surgery and hip replacement [6]. The determination of whether the femoral head collapses and the degree of articular cartilage collapse is an important guiding basis for clinical treatment [7, 8]. Therefore, imaging is often used in clinical examination and prediction, among which CT and X-ray scanning are commonly used [9]. X-ray scanning, as one of the conventional methods for the diagnosis of ONFH, mainly reflects the results of disease examination by the tissue absorption rate of the X-ray; however, it is not sensitive to the early lesions of ONFH [10]. CT scanning, which is more detailed than an X-ray examination, has high sensitivity and contrast and can display well the collapse and subchondral fractures. As a routine clinical diagnosis and treatment of ONFH, CT and X-ray scanning have a high frequency of use, good popularization, and advantages that other methods do not have [11]. Since there is no unified conclusion on the prediction of the femoral head collapse before replacement at this stage, it will be further studied in this study.

RETRACTED

To make the research more representative, the medical big data samples were collected and analyzed. Medical big data have the characteristics of a large amount of data, fast growth, variety, and high value [12]. To analyze and process the big data in this study more effectively, the data mining algorithm was used to classify and process the medical big data. Among them, the decision tree algorithm is the most commonly used technology in data mining classification. However, because of the high complexity of generating fuzzy rules and the poor stability of global modeling, a heuristic swarm intelligence optimization algorithm was used—grey wolf optimization (GWO)—to process the decision tree algorithm [13].

In this study, the effect of the CT and X-ray examinations before the hip replacement to predict the collapse of the necrotic femoral head in the context of medical big data based on the classification of the decision tree algorithm of the difference GWO was studied and analyzed to provide a more effective examination basis for the formulation of treatment plans for patients with ONFH.

## 2. Related Works

According to clinical treatment experience, the reasonable and accurate staging of ONFH has a significant impact on the determination of surgical scheme, treatment effect, and prognosis [14]. Reasonable and accurate staging will affect the formulation of treatment plans. At present, imaging examinations are used to diagnose the stage of the femoral head and check the collapse, and they are used to guide the formulation of the surgical plan. A large number of studies showed that the X-ray and CT examinations have good diagnostic effects in the staging of the femoral head and the diagnosis of collapse. The correlation research of the femoral neck fracture reduction quality and femoral head necrosis biomechanics of Wang et al. [15], the research of core decompression or femoral muscle pedicle bone graft in the treatment of nontraumatic femoral head necrosis of Li et al. [16], and about SPECT/CT in the prediction of the femoral neck fracture osteonecrosis in the study of the diagnostic value of Yoon et al. [17] reflect the X-ray and CT examinations in the diagnosis and treatment of ONFH disease. In line with the results of this study, the staging results of the X-ray and CT examinations with the measurement results of a solid bone were compared in this study. The results showed that the diagnostic sensitivity, specificity, and accuracy of the two methods reached more than 90%, and the consistency Kappa value of the diagnostic results reached more than 0.65, which fully reflected the good application effect of the X-ray and CT examinations in ONFH staging. This study also concluded that there was no significant difference between the X-ray and CT examination in the detection of femoral head collapse degree and the measurement results of a solid bone. For example, there was no significant difference between the X-ray measurement results *a*′ (22.39 ± 1.98) mm, *b*′ (23.99 ± 2.28) mm, and *c*′ (24.11 ± 1.88) mm and the solid measurement results *a* (22.43 ± 2.01) mm, *b* (24.03 ± 2.12) mm, and *c* (24.22 ± 2.48) mm in X group (*P* > 0.05). The CT group was the same. It is consistent with the research results on the dynamic evolution of bone structure and the risk of dynamic collapse of the femoral head necrosis by the CT of Huang et al. [18]. Ding et al. [19] used the results of the X-ray examination to determine the treatment plan in the study of individual extracorporeal shock wave therapy for early ONFH, and the results showed that the condition of patients with ONFH improved significantly.

RETRACTED

To make the research more comprehensive and extensive, this study takes patients nationwide as the research objects to carry out the related research, which involves the application of medical big data. The analysis of the research data becomes difficult. Therefore, it is important to do a good job of intelligent classification of medical big data in advance. In this study, a decision tree algorithm based on the difference GWO was used to carry out the intelligent classification of medical big data, and the performance of its application was compared. The results show that the accuracy (0.722), TPR (0.849), FPR (0.201), and *F*_1_-score (0.758) improved. It is consistent with the research of Supriya and Deepa [20] on a new method for breast cancer prediction based on the neural network classifier optimized in a big data environment. It is also consistent with the research of Gao and Zhao [21] on an improved variable weight GWO algorithm, suggesting that the GWO algorithm has a good application prospect [22].

## 3. Research Process

### 3.1. Medical Big Data Classification Algorithm Based on Difference GWO Decision Tree

#### 3.1.1. GWO Algorithm

The GWO algorithm is established on the basis of the grey wolf hierarchy and hunting rules in nature. There are four grades of wolf groups, and the grade from high to low is as follows: leader-*α*, subordinate-*β*, executor-*δ*, and follower-*ω*. In the optimization process of the GWO algorithm, the advantages and disadvantages of the calculation results are the basis of *α*, *β*, *δ*, and *ω* corresponding to the other solutions. The three stages of the wolves' predation process are tracking, hunting, and attacking. They can be separately defined in mathematics as follows:

The first is the tracking stage. During the predation process, the behavior of the tracking prey can be expressed as follows:

(1) $$\begin{array}{c} \overset{⟶}{I}=\overset{⟶}{G}\cdot \overset{⟶}{M_{b}}\left(x\right)-\overset{⟶}{M}\left(x\right),\\ \overset{⟶}{M}\left(x+1\right)=\overset{⟶}{M_{b}}\left(x\right)-\overset{⟶}{F}\cdot \overset{⟶}{I}, \end{array}$$

in which $\overset{⟶}{M_{b}}$ is the position vector of the prey. $\overset{⟶}{M}$ is the position vector of the wolves. $\overset{⟶}{I}$ is the position vector distance between the prey and the wolves. *x* is the current number of iterations. $\overset{⟶}{G}$ and $\overset{⟶}{F}$ are the collaborative coefficient vectors that an be expressed as follows:

(2) $$\begin{array}{c} \overset{⟶}{G}=2\cdot \overset{⟶}{h_{2}},\\ \overset{⟶}{F}=2\overset{⟶}{e}\cdot \overset{⟶}{h_{1}}-\overset{⟶}{e}. \end{array}$$

in which $\overset{⟶}{h_{1}}$ and $\overset{⟶}{h_{2}}$ are the one-dimensional random vectors, and the interval is [0, 1]. $\overset{⟶}{e}$ refers to the coefficient vector, with the increase of the number of iterations from 2 to 0 linear decline.

The second stage is the pursuit stage. In this stage, the optimal solution position in the iterative process is unknown. Therefore, it is necessary to consider the positions of three potential solutions *α*, *β*, and *δ* in the mathematical expression. Details are as follows:

(3) $$\begin{array}{c} \overset{⟶}{I_{\alpha }}=\overset{⟶}{G_{1}}\cdot \overset{⟶}{M_{\alpha }}-\overset{⟶}{M},\\ \overset{⟶}{I_{\beta }}=\overset{⟶}{G_{2}}\cdot \overset{⟶}{M_{\beta }}-\overset{⟶}{M},\\ \overset{⟶}{I_{\delta }}=\overset{⟶}{G_{3}}\cdot \overset{⟶}{M_{\delta }}-\overset{⟶}{M},\\ \overset{⟶}{M_{1}}=\overset{⟶}{M_{\alpha }}-\overset{⟶}{F_{1}}\cdot \overset{⟶}{I_{\alpha }},\\ \overset{⟶}{M_{2}}=\overset{⟶}{M_{\beta }}-\overset{⟶}{F_{2}}\cdot \overset{⟶}{I_{\beta }},\\ \overset{⟶}{M_{3}}=\overset{⟶}{M_{\delta }}-\overset{⟶}{F_{3}}\cdot \overset{⟶}{I_{\delta }},\\ \overset{⟶}{M}\left(x+1\right)=\frac{\overset{⟶}{M_{1}}+\overset{⟶}{M_{2}}+\overset{⟶}{M_{3}}}{3}. \end{array}$$

Finally, the attack stage of predation: ending hunting and obtaining the optimal solution. In the mathematical sense, the decreasing of $\overset{⟶}{e}$ indicates that the closer to the prey, the smaller the fluctuation range *F* ∈ [−*e*, *e*]. When $\overset{⟶}{e}$ reduces from 2 to 0, if |*F*| ≤ 1, then it indicates the wolves are close to the prey. If |*F*| > 1, it means the wolves are far away from the prey. The algorithm will only obtain the local optimal solution, thus losing the optimal solution position, and $\overset{⟶}{e}$ is expressed as follows:

(4) $$\begin{array}{c} e=2-\frac{2x}{{\text{Iter}}_{\max}}, \end{array}$$

where Iter_max_ is the maximum number of iterations.

RETRACTED

#### 3.1.2. Decision Tree Algorithm Based on Difference GWO

To solve the problem of data imbalance and data type missing in the big data classification, the weight of the data category is modified as the research focus. The construction of the decision tree can be divided into three processes, namely feature selection, decision tree generation, and decision tree pruning [3].

Feature selection, in general, is based on the information gain theory. The information gain theory can provide a standard for decision making. By calculating the information gain of each data feature, the feature with the largest information gain is selected. The specific algorithm is as follows:

(5) $$\begin{array}{c} \text{Gain}\left(S,R_{p}\right)=Q\left(S\right)-Q_{R_{p}}\left(S\right), \end{array}$$

in which*R*_*p*_ refers to the sample features, *S* refers to the training set, and *Q* refers to each decision node candidate attribute list.

(6) $$\begin{array}{c} Q\left(S\right)=-\sum_{j=1}^{k}\frac{k\left(B_{j}\cdot S\right)}{\left|S\right|}\log^{2}\frac{k\left(B_{j}\cdot S\right)}{\left|S\right|},\\ Q_{R_{p}}\left(S\right)=\sum_{u\in C\left(R_{p}\right)}\frac{\left|S_{u}^{R_{p}}\right|}{\left|S\right|}Q\left(S_{u}^{R_{p}}\right), \end{array}$$

in which *k*(*B*_*j*_ · *S*) refers to the number of objects of *B*_*j*_ in the training set *S*. *C*(*R*_*p*_) refers to the finite field of features *R*_*p*_. |*S*_*u*_^*R*_*p*_^| refers to the cardinality of the object set whose feature *R*_*p*_ value is *u*. The information gain ratio is expressed as follows:

(7) $$\begin{array}{c} \text{Gro}\left(S,R_{p}\right)=\frac{\text{Gain}\left(S,R_{p}\right)}{\text{SplitInfo}\left(S,R_{p}\right)}, \end{array}$$

in which SplitInfo(*S*, *R*_*p*_) refers to the potential information generated by dividing *Q* into *n* subsets. The expression is as follows:

(8) $$\begin{array}{c} \text{SplitInfo}\left(S,R_{p}\right)=\sum_{u\in C\left(R_{p}\right)}\frac{\left|S_{u}^{R_{p}}\right|}{\left|S\right|}\log^{2}\frac{\left|S_{u}^{R_{p}}\right|}{\left|S\right|}. \end{array}$$

The generation of the decision tree: the calculation in this part starts with the root node, and the maximum feature is selected from all the potential information gain at node *Q* as the node feature. Then, the child nodes are constructed according to the value of the feature and recursive based on the above calculation method. The mark of the completion of the decision tree construction is that the information gain of all features is small or no feature can be selected.

RETRACTED

The pruning of the decision tree: by optimizing the loss function to remove the meaningless classification features and reduce the overall complexity of the algorithm, it is usually realized by minimizing the overall loss function of the decision tree. The expression of the loss function is as follows:

(9) $$\begin{array}{c} C_{a}\left(T\right)=C\left(T\right)+a\left|T\right|, \end{array}$$

in which *T* refers to any subtree, |*T*| refers to the number of subtree nodes, *C*(*T*) refers to the prediction error of training data, and *a* refers to the parameters that measure the fitting degree of computational complexity and training data.

Optimization method: the decision tree classifier is optimized by the difference grey wolf algorithm, and the accuracy of the classifier is taken as the objective function to optimize and modify the weight of the data category to construct a better decision tree. The optimized objective function is as follows:

(10) $$\begin{array}{c} \text{OB}=\text{max}\left(\text{accuracy}\right), \end{array}$$

in which accuracy is the accuracy of the classifier. However, the GWO algorithm also has some limitations, such as high complexity and lack of optimal solution search ability. Therefore, on the basis of the conventional GWO algorithm, equation (3) of the potential solution position is updated as follows:

(11) $$\begin{array}{c} \overset{⟶}{M}\left(x+1\right)=\left[\frac{\overset{⟶}{M_{1}}+\overset{⟶}{M_{2}}+\overset{⟶}{M_{3}}}{3}\right]+\left[\frac{\overset{⟶}{M_{1}^{\prime }}+\overset{⟶}{M_{2}^{\prime }}+\overset{⟶}{M_{3}^{\prime }}}{3}\right]. \end{array}$$

Here, $\overset{⟶}{M_{1}^{\prime }}$, $\overset{⟶}{M_{2}^{\prime }}$, and $\overset{⟶}{M_{3}^{\prime }}$ are the first, second, and third worst solutions.

RETRACTED

#### 3.1.3. Evaluation Indicators

The performance evaluation indexes of the classification algorithm are evaluated by accuracy (Acc), true positive rate (TPR), false positive rate (FPR), and *F*_1_-score.

There are only positive and negative values in the two classification problems. Then, the calculation expressions of Acc, TPR, FPR, and *F*_1_-score are as follows:

(12) $$\begin{array}{c} \text{Acc}=\frac{\text{TP}+\text{TN}}{\text{TP}+\text{TN}+\text{FP}+\text{FN}},\\ \text{TPR}=\frac{\text{TP}}{\text{TP}+\text{FN}},\\ \text{FPR}=\frac{\text{FP}}{\text{FP}+\text{TN}},\\ F_{1}-\text{score}=\frac{2\times \text{TP}}{2\times \text{TP}+\text{FP}+\text{FN}}. \end{array}$$

### 3.2. Research Objects

In this study, a retrospective study was conducted on the selection of research samples nationwide. A total of 152,000 patients with ONFH and hip replacement were selected in the tertiary hospitals from January 2019 to January 2021. There were 98,100 male patients and 53,900 female patients, aged between 30 years to 70 years, with an average age of (51.22 ± 19.08) years. There were 112,000 patients in stage III and 40,000 patients in stage IV. According to the random number method, all patients were divided into two groups. The X-ray examination results of the patients were the study sample (X group), and the CT examination results of patients were the study sample (CT group), with 76,000 patients in each group. The actual measurement results of the femoral head after the hip replacement were used as the gold standards to evaluate the effect of the two groups of detection methods. The study was approved by the medical ethics committee.

Inclusion criteria: (a) the diagnosis of the unilateral avascular necrosis of the femoral head before the hip replacement and the FICAT stage are stages III and IV [23]. (b) Unilateral total hip arthroplasty was performed. (c) X-ray (pelvic position and frog position) and CT (double hip CT scan) were used for scanning within one week before the operation. (d) Patients and their families were informed, and they agreed.

Exclusion criteria: (a) patients with infection, (b) patients with tuberculosis, (c) patients with tumor diseases, (d) patients with severe osteoporosis, and (e) patients with incomplete X-ray or CT scan results.

### 3.3. Requirements for X-Ray and CT Scanning

X-ray and CT scanning positions: both the standard abduction neutral position-anterior median line and the lower limbs were at an angle of 15°, and the feet were placed perpendicularly to the horizontal plane. X-ray examination should also maintain the pelvic position.

During the examination, the patient was supine on the examination bed, aligning the centerline of the body with the centerline of the examination bed and placing the lower limb straight. The anterior superior iliac spine should be equidistant from the bed surface. In order to maintain the consistency of the center of the femoral head, it is necessary to wear “Ding” shoes to fix the lower limbs during the examination.

RETRACTED

### 3.4. Measurement Method

#### 3.4.1. Measurement Method of Solid Femoral Head

The pathological femoral head was resected during the operation was washed with normal saline. The femoral head that has not been completely resected is approximately spherical. The surgical incision is longitudinal, and the coronal surface is round. The specific measurement methods are as follows:

  Step 1: the femoral head was cut from the median along the coronal plane with an electric pendulum saw to expose the coronal plane of the femoral head, as shown in Figure 1(a).
  Step 2: in the coronal plane of the femoral head, drawing tools were used (such as compasses, triangles, and angle measuring device) to determine the center of the femoral head of this circular coronal plane (*D*), as shown in Figure 1(b).
  Step 3: a line (*X*) was drawn connecting the femoral neck and the apex of the femoral head, passing through the center (*D*), and a line (*Y*) passing through the center and perpendicular to the line (*X*) was drawn, as shown in Figure 1(c).
  Step 4: the distance from the center of the circle (*D*) on the line (*X*) to the apex of the femoral head was set as *a*, and the distance from the center of the circle (*D*) on the line (*Y*) to the apex of the lateral femoral head was set as *b*. Finally, the angles between *c* and *a*, *c* and *b* are determined to be 45°, as shown in Figure 1(d).

Among them, *a*, *b*, and *c* represented the actual height of lateral, medial, and middle of the femoral head after collapsing.

#### 3.4.2. Imaging Data Measurement

Image measurement and analysis software DigimizerV3.8.1 (Med Cale Software, USA) was used to measure the actual height of the lateral, medial, and middle femoral head after the X-ray examination and CT scan. The measurement method was consistent with the measurement method of the solid bone. The height of the lateral, medial, and middle femoral head after the X-ray examination was expressed as *a*′, *b*′, and *c*′, respectively, as shown in Figure 2(a), and the height of the lateral, medial, and middle femoral head after the CT scan was expressed as *a*″, *b*″, and *c*″, respectively, as shown in Figure 2(b).

### 3.5. Observation Indicators

By comparing with the measurement results of the solid femoral head, the sensitivity, specificity, and diagnostic accuracy of the two groups of the inspection methods for the femoral head collapse were analyzed, as shown in Table 1. The Kappa value was calculated by analyzing the diagnostic consistency of the X-ray and CT examinations for the femoral head collapse. If Kappa = 1, the diagnostic results were completely consistent. If Kappa = −1, the diagnostic results were completely inconsistent. Kappa ≥ 0.75, suggesting that the consistency of diagnosis was quite satisfactory. Kappa < 0.4, suggesting that the consistency of the diagnostic results was not ideal.

RETRACTED

### 3.6. Statistical Method

SPSS22.0 statistical software was used to analyze the data. The measurement data in line with normal distribution were expressed as mean ± standard deviation ($\bar{x}$ ± *s*), and the two decimals were retained. The paired *t*-test was used for comparison in the group, and the independent sample *t*-test was used for comparison between the two groups. The quantitative data conforming to the skewness distribution were represented by the median (range), and the comparison between the two groups was tested by the Wilcoxon rank-sum test. The enumeration data were expressed as a percentage (%), and one decimal was retained. The comparison between the two groups was conducted using the continuity correction of the *χ*^2^ test or *χ*^2^ test. The *P* value retained three decimal places, and *P* < 0.05 indicated that the difference was statistically significant.

## 4. Results

### 4.1. Detection Results of Algorithm Performance

Figure 3 is the classification performance test results of the difference GWO decision tree algorithm and other algorithms used in this study. The accuracy (0.722), TPR (0.849), FPR (0.201), and *F*_1_-score (0.758) of the difference GWO decision tree algorithm improved compared with the scale-free binary particle swarm optimization (SFBPSO) and the simple GWO algorithm [23].

### 4.2. Comparison of General Data of Patients

According to the statistics of the general treatment of patients in terms of gender distribution, there were 50,500 male patients (51.48%) and 27,400 female patients (50.83%) in the X group. There were 47,600 male patients (48.52%) and 26,500 female patients (49.17%) in the CT group with no significant difference (*P* > 0.05). In terms of age distribution, the average age of patients in the X group was (50.39 ± 18.98) years and that in the CT group was (51.41 ± 19.01) years with no significant difference (*P* > 0.05). In terms of the FICAT staging distribution, there were 54,100 patients with stage III and 20,100 patients with stage IV in the X group and 57,900 patients with stage III and 19,900 patients with stage IV in the CT group, and there was no significant difference (*P* > 0.05), as shown in Figure 4. The above comparison suggests that the two groups of comparisons in this study are comparable.

RETRACTED

### 4.3. Statistics of Measurement Results

Figure 5 shows the mean values of the X-ray measurement results and the corresponding lateral, medial, and intermediate heights of the solid femoral head after collapse in the X group. The mean values of the X-ray measurement results *a*′, *b*′, and *c*′ were (22.39 ± 1.98) mm, (23.99 ± 2.28) mm, and (24.11 ± 1.88) mm, respectively. The mean values of *a*, *b*, and *c* measured by the solid femoral head were (22.43 ± 2.01) mm, (24.03 ± 2.12) mm, and (24.22 ± 2.48) mm, respectively. There was no significant difference (*P* > 0.05).  Figure 6 is the measurement schematic of the X group.  Figure 7 shows the mean values of the lateral, medial, and intermediate heights of the CT scan measurement results and the corresponding solid femoral head after collapse in in the CT group. The mean values of the CT ray measurement results *a*″, *b*″, and *c*″ are (22.33 ± 1.98) mm, (24.01 ± 2.18) mm, and (24.21 ± 1.89) mm, respectively. The mean values of *a*, *b*, and *c* of the measurement results of the solid femoral head were (22.45 ± 2.11) mm, (24.11 ± 2.13) mm, and (24.12 ± 2.42) mm, respectively, and there was no significant difference in the comparison (*P* > 0.05).  Figure 8 shows the measurement schematic of patients in the CT group.

### 4.4. Statistics of Staging Results

Table 2 shows the statistics of the X-ray measurement results and the solid femoral head measurement staging results of the X group, and Table 3 shows the statistics of the CT scanning measurement results and solid femoral head measurement staging results of the patients in the CT group. The X-ray examination and CT scanning measurement results and the solid bone measurement results of the patients in stage III and stage IV of the two groups were statistically analyzed.

### 4.5. Comparison of Diagnostic Effect

According to the above diagnostic results, the diagnostic sensitivity, specificity, accuracy, and consistency of the two groups were calculated. The diagnostic sensitivity, specificity, accuracy, and consistency of stage III patients in the X group were 97.92%, 93.67%, 97.52%, and 0.69, respectively. The diagnostic sensitivity, specificity, accuracy, and consistency of stage IV patients were 94.96%, 94.09%, 94.88%, and 0.71, respectively. The diagnostic sensitivity, specificity, accuracy, and consistency of stage III patients in the CT group were 97.24%, 91.96%, 96.75%, and 0.68, respectively. The diagnostic sensitivity, specificity, accuracy, and consistency of stage IV patients were 97.70%, 93.98%, 97.24%, and 0.72, respectively.

RETRACTED

Figure 9 is the comparison of the diagnostic results in stage III, and Figure 10 is the comparison of stage IV diagnostic effects. By the above experimental results, it can be observed that there was no significant statistical difference in the sensitivity, specificity, accuracy, and consistency of the diagnosis results of stage III and stage IV between the two groups (*P* > 0.05), as shown in Figures 9 and 10.

## 5. Conclusion

This study studies and analyzes the effect of the CT and X-ray examinations before the hip replacement to predict the collapse of the necrotic femoral head under the background of medical big data based on the difference GWO decision tree algorithm classification. The results showed that the measurement results of the X-ray and CT before the hip replacement are highly consistent with those of the solid femoral head specimens, which could effectively predict the collapse of the femoral head necrosis and accurately stage it. However, this study has the problem of an imperfect index setting, such as not comparing it with the measurement results of a healthy femoral head. However, the study can fully reflect the X-ray and CT examinations in the diagnosis of the ONFH disease and has good application prospects that are worthy of clinical promotion.

## Figures and Tables

**Figure 1:** Measurement method of solid femoral head.

**Figure 2:** Imaging data measurement schematic.

**Figure 3:** Classification performance comparison of algorithms.

**Figure 4:** Distribution of FICAT staging.

**Figure 5:** Measurement results of X group.

**Figure 6:** Measurement schematic of X group. (a) X-ray and (b) solid bone.

**Figure 7:** Measurement results of CT group.

**Figure 8:** Measurement schematic of CT group. (a) CT and (b) solid bone.

**Figure 9:** Comparison of diagnostic results in stage III: (a) sensitivity, specificity, accuracy, and (b) consistency.

**Figure 10:** Comparison of stage IV diagnostic effects: (a) sensitivity, specificity, accuracy, and (b) consistency.

**Table 1:** Calculation methods of diagnostic sensitivity, specificity, and accuracy.

Indicator	Calculation methods
Sensitivity	Patients with actual illness and correct diagnosis/total patients × 100%
Specificity	Actual disease-free and correctly diagnosed patients/total patients × 100%
Accuracy	(Number of patients diagnosed in the affected population + number of patients diagnosed in the nonaffected population)/total patients × 100%

**Table 2:** Diagnosis results of X group.

		Measurement results of solid bone (*n* = 54,100)		Total
		Stage III	Nonstage III	
X-ray measurement results (*n* = 54,100)	Stage III	48,010	320	48,330
	Nonstage III	820	4750	5770
Total		49,030	5070	54,100

		Measurement results of solid bone (*n* = 20,100)		Total
		Stage IV	Nonstage IV	
X-ray measurement results (*n* = 20,100)	Stage IV	17,320	110	7430
	Nonstage IV	920	1750	2670
Total		18,240	1860	20,100

RETRACTED

**Table 3:** CT diagnosis results.

		Measurement results of solid bone (*n* = 57,900)		Total
		Stage III	Nonstage III	
CT scan measurement results (*n* = 57,900)	Stage III	51,100	430	51,530
	Nonstage III	1450	4920	6370
Total		52,550	5350	57,900

		Measurement results of solid bone (*n* = 19,900)		Total
		Stage IV	Nonstage IV	
CT scan measurement results (*n* = 19,900)	Stage IV	17,010	150	17,160
	Nonstage IV	400	2340	2740
Total		17,410	2490	19,900

## Data Availability

The simulation experiment data used to support the findings of this study are available from the corresponding author upon request.

## References

[1] Zhao D., Zhang F., Wang B. (2020). Guidelines for clinical diagnosis and treatment of osteonecrosis of the femoral head in adults (2019 version). *Journal of Orthopaedic Translation*.

[2] Liu L.-H., Zhang Q.-Y., Sun W., Li Z.-R., Gao F.-Q. (2017). Corticosteroid-induced osteonecrosis of the femoral head. *Chinese Medical Journal*.

[3] Chen G., Zhong L., Wang Q. (2019). The expression of chondrogenesis-related and arthritis-related genes in human ONFH cartilage with different Ficat stages. *PeerJ*.

[4] Wu X., Sun W., Tan M. (2019). Noncoding RNAs in steroid-induced osteonecrosis of the femoral head. *BioMed Research International*.

[5] Zhang X., You J. m., Dong X. j., Wu Y. (2020). Administration of mircoRNA‐135b‐reinforced exosomes derived from MSCs ameliorates glucocorticoid‐induced osteonecrosis of femoral head (ONFH) in rats. *Journal of Cellular and Molecular Medicine*.

[6] Zhou W., Qu M., Lv Y., Zhu J. (2019). New advances in stem cell therapy for osteonecrosis of the femoral head. *Current Stem Cell Research and Therapy*.

[7] Li T. x., Huang Z. q., Li Y. (2019). Prediction of collapse using patient‐specific finite element analysis of osteonecrosis of the femoral head. *Orthopaedic Surgery*.

[8] Hatanaka H., Motomura G., Ikemura S. (2019). Differences in magnetic resonance findings between symptomatic and asymptomatic pre-collapse osteonecrosis of the femoral head. *European Journal of Radiology*.

[9] Feng S., Li B., Li G. (2020). Abnormal spatial patterns of intrinsic brain activity in osteonecrosis of the femoral head: a resting-state functional magnetic resonance imaging study. *Frontiers in Human Neuroscience*.

[10] Zeng J., Zeng Y., Wu Y., Liu Y., Xie H., Shen B. (2020). Acetabular anatomical parameters in patients with idiopathic osteonecrosis of the femoral head. *The Journal of Arthroplasty*.

RETRACTED

[11] Zhu L., Han J., Guo R. (2020). An automatic classification of the early osteonecrosis of femoral head with deep learning. *Current Medical Imaging*.

[12] Lv Z. H., Liang Q. (2020). Analysis of healthcare big data. *Future Generation Computer Systems*.

[13] Chakraborty S., Pradhan R., Ashour A. S., Moraru L., Dey N. (2020). Grey-wolf-based Wang’s demons for retinal image registration. *Entropy*.

[14] Hua K.-c., Yang X.-g., Feng J.-t. (2019). The efficacy and safety of core decompression for the treatment of femoral head necrosis: a systematic review and meta-analysis. *Journal of Orthopaedic Surgery and Research*.

[15] Wang Y., Ma J. x., Yin T. (2019). Correlation between reduction quality of femoral neck fracture and femoral head necrosis based on biomechanics. *Orthopaedic Surgery*.

[16] Li M., Li D., Liu P., Zhang Y., Ma L., Xu F. (2016). Core decompression or quadratus femoris muscle pedicle bone grafting for nontraumatic osteonecrosis of the femoral head: a randomized control study. *Indian Journal of Orthopaedics*.

[17] Yoon J. Y., Lee S. J., Yoon K. S., Yoon P. W. (2020). The diagnostic value of SPECT/CT in predicting the occurrence of osteonecrosis following femoral neck fracture: a prospective cohort study. *BMC Musculoskeletal Disorders*.

[18] Huang Z., Tan B., Ye H., Fu F., Wang R., Chen W. (2020). Dynamic evolution of osseous structure in osteonecrosis of the femoral head and dynamic collapse risks: a preliminary CT image study. *Journal of Orthopaedic Surgery and Research*.

[19] Ding H., Wang S., Feng H. (2019). Clinical efficacy of individual extracorporeal shockwave treatment. *Der Orthopäde*.

[20] Supriya M., Deepa A. J. (2020). A novel approach for breast cancer prediction using optimized ANN classifier based on big data environment. *Health Care Management Science*.

[21] Gao Z. M., Zhao J. (2019). An improved grey wolf optimization algorithm with variable weights. *Computational Intelligence and Neuroscience*.

[22] Plonka A., Urban I., Wang H.-L. (2018). Decision tree for vertical ridge augmentation. *The International Journal of Periodontics and Restorative Dentistry*.

[23] Kolk A., Neff A. (2015). Long-term results of ORIF of condylar head fractures of the mandible: a prospective 5-year follow-up study of small-fragment positional-screw osteosynthesis (SFPSO). *Journal of Cranio-Maxillofacial Surgery*.

